# Analysis of the Running Ability Mining Model of Football Trainers Based on Dynamic Incremental Clustering Algorithm

**DOI:** 10.1155/2022/3255886

**Published:** 2022-06-29

**Authors:** Peng Zhao, Fei Xue, Xipeng Zhang

**Affiliations:** ^1^University Physical Education Department, Huanghai University, Qingdao, Shandong 266427, China; ^2^School of Preschool Education, Huanghai University, Qingdao, Shandong 266427, China

## Abstract

Fast-running ability is a very important basic quality of football players. However, players are dynamic. It is difficult for coaches to grasp the running speed, instantaneous acceleration, and other indicators of small athletes in real time with the naked eye. Therefore, to accurately test the performance of athletes in fast-running ability, this paper studies the running ability mining model of football coaches based on the dynamic incremental clustering algorithm. According to scientific procedures and methods, the evaluation model and standard of running ability of Chinese elite female football players are established. The effectiveness of the model is 0.83, as verified by the standard recognition method, which shows that the evaluation model is efficient. The research considers the denoising of the original data. The model has rich data and standard test methods and procedures. It can be used as a measure of the running ability of China's elite female football players in a certain period and range. The research solves the problem of the insufficient running ability of domestic football players. It provides an important reference for training the next generation of excellent national football players.

## 1. Introduction

Football is a high-intensity, intermittent sport, which requires athletes' aerobic and anaerobic endurance and explosive speed to be very high. Many coaches believe that athletes' running ability has become one of the important factors for the team to win in the competition [1, 2]. It is the core method to study the physical ability of a football match to evaluate the running ability of players in the football match. From the early manual notation method, game video analysis method, radio telemetry, and GPRS technology, it has been developed to the current analysis method using computer video technology. Hence, the analysis method of computer video technology is the mainstream in this field [3]. The fast-running ability is a very important basic quality of football players. The fast-running ability of football players includes the fast-starting ability, short-distance sprint ability, fast-changing direction ability, fast-turning and running ability, etc. Under normal circumstances, football trainers quantify the outside of football players' running ability training, mainly through the analysis of video and GPS positioning technology to track the running distance and running speed of football players [4, 5]. The basic feature of football running is the position characteristics of players on the field. For example, there is a huge difference between the running of forward players and middle and backcourt players. However, from the current research results, there is a lack of special research and evaluation on the running of players in different positions [6].

In the process of football training and running, the coach hopes to discover the small players of different sports types and find the hidden index characteristics that cannot be discovered by the naked eye. However, the movement of players is dynamic, and it is difficult for coaches to grasp the running speed, instantaneous acceleration, and other indicators of small players in real time with the naked eye. Therefore, how to mine and analyze the collected acceleration of small players based on the application of existing intelligent collection technology in football training data using the dynamic incremental clustering algorithm in data mining to deeply and objectively reflect the technical and tactical categories and comprehensive strength of each player is the problem to be studied in this paper [7, 8]. Although each incremental clustering algorithm has certain limitations, on the whole, incremental clustering inherits the execution results of existing clustering. Through the processing of new data one by one or in batch, it largely avoids a large number of repeated calculations, reduces the amount of calculation, saves system expenses, and improves the clustering efficiency. Especially when the amount of data is larger, incremental clustering can better reflect its advantages [9]. Traditional clustering algorithms are aimed at static datasets, however, they cannot deal with the dynamic data that is updated and changed at any time efficiently. Therefore, the incremental clustering algorithm came into being. On the basis of the original clustering results, for the new dataset, analyze the relationship and influence between the new dataset and the original clustering results, and use the incremental clustering algorithm to overlay them to obtain the final clustering results, which avoids the repeated calculation of a large number of original datasets and greatly improves the efficiency [10, 11].

Static clustering mining is carried out on the data recorded by naked eyes when watching football videos. This kind of research is done only by watching the analysis videos after the game and depends entirely on the judgment of naked eyes. It has a serious lag, and a large amount of hidden information cannot be discovered by naked eyes. Hence, it cannot truly reflect the training technical indicators in real time. Therefore, it is necessary to collect, mine, and analyze athletes' training running data in real time and then analyze their technical and tactical types. Fast-starting ability is the ability of athletes to quickly change from a static state to a running state. The importance of fast-starting ability in football based on the dynamic incremental clustering algorithm even exceeds the maximum speed of athletes. Players with good starting ability can easily get rid of their opponents and take the lead in various technical links, such as catching the ball, passing, stealing, and making up the position [12, 13]. The dynamic incremental clustering algorithm is used to mine and analyze potentially hidden important information from a large number of complicated data on football trainers' running ability. The clustering algorithm is to mine the similarity between data according to data characteristics and cluster the similar data into one class. Short-distance sprint ability is a special quality that football players must possess. It not only requires the athletes to have the ability to run quickly in short distances but also requires them to have the ability to carry on continuously. In football competition based on the dynamic incremental clustering algorithm, the requirement of practice is the focus of the training class [14, 15]. If we want to completely change the current problem of the insufficient running ability of domestic football players, we must start with the football players in the youth stage, solve the problem of insufficient running ability of Chinese football players from the youth stage, and train the next generation of outstanding national football players, which is an important link for the long-term development of Chinese football. On the basis of sorting out the existing research results, this study screens the existing evaluation indexes, and the ultimate goal is to establish the evaluation model of athletes' running ability in different positions to provide the basis for training and competition monitoring.

## 2. Related Work

Chalmers et al. put forward that the ability of sprint is the core physical quality of forward athletes and the key factor determining the level of forward athletes. Middle- and short-distance sprint and continuous round-trip sprint are the typical running characteristics of forwards. The total distance of high-speed running and competition running can evaluate its activity range and ability [16]. Prager et al. proposed that athletes jog in place. Look at the coach's gesture and start quickly. Pay attention not to use passwords but to use gestures to enhance the athletes' observation and response ability, which is more combined with the actual situation of the game [17]. West et al. put forward that in modern football matches, the requirements for forwards are higher. In addition to having efficient scoring ability, the ability to connect with avant-garde players in attack, involve defensive players and create scoring opportunities for avant-garde players should also be improved accordingly. Therefore, we see more goals from avant-garde players, which are related to the running of avant-garde players in the game [18]. Sheng et al. proposed that China is a powerful country in sports but not in football. With the development of football, China's attention to football has also risen to the national level. General Secretary Xi put forward the lofty dream of “holding the world cup, entering the World Cup finals, and winning the world cup champion” [19]. Azarkasb et al. put forward that football is a high-intensity and intermittent sport, which has very high requirements for athletes' aerobic and anaerobic endurance and explosive speed. Many coaches believe that the running ability of athletes has become one of the important factors for the team to win in the game [20]. Zhang et al. proposed that the research results obtained through the research on the running distance characteristics of domestic excellent young football players can provide data reference for the development of Chinese young football, facilitate the coach team to formulate reasonable training plans according to the data, train for everyone, and greatly improve the overall running ability of each player [21]. Meylan et al. pointed out that to fundamentally change the present situation of Chinese football, more scientific guidance is needed to change and develop football. Therefore, the development of Chinese football should still look at the problem from a long-term perspective. On the basis of developing and cultivating active football players, we also need to vigorously develop and cultivate the next generation of Chinese football players, attach importance to the training of young football players, give them the most scientific guidance and systematic training, and provide more opportunities to communicate with foreign football when their football level is still rising [22]. Hedlund et al. put forward that avant-garde players are the link and bridge between the frontcourt and the backcourt, and they should constantly participate in attack and defense. Hence, their range of activities is also an important indicator, and the total running distance of the game is an important embodiment of their range of activities [23]. Conine et al. puts forward that FIFA will expand the number of participating teams that can enter the finals of the World Cup from the current 32 to 48 teams from the 2026 World Cup to meet the needs of the development of football all over the world. This move also greatly encourages the development of football in various countries, greatly enhances people's love, and better proves that football is the “first sport in the world” [24]. Rusliani et al. put forward that it is impossible to improve the running ability of football players at the national team level again. Hence, we should focus more on the level of young football players, who are in a stage of rising both physically and psychologically. At this stage, if enough attention is paid to their running ability, then their running ability will have a qualitative leap compared with that of active football players [25, 26].

This paper studies the running ability of football trainers based on the dynamic incremental clustering algorithm. The dynamic incremental clustering algorithm hopes to assist coaches to find the technical and tactical categories of small players. At the same time, the clustering sample is a three-dimensional acceleration index. There is no problem of different density caused by a wide variety of clustering sample data. Therefore, it is most appropriate to select the mean algorithm in the clustering algorithm. Many athletes jog forward together and watch the coach's gestures move forward, backward, left, and right quickly. Pay attention to the coach's gestures. When changing direction, avoid other team members. It is more difficult for many people to practice at the same time. When avoiding other team members, there should be changing direction and dodging. However, because of the large amount of training running data and real-time change and update, the complexity of the algorithm should not be too high, which is difficult to be met by many classical clustering algorithms. Through the research and analysis of the highest level youth football match in China, the research findings from theoretical data to data will provide a strong reference basis for their coaches in running ability training. This research belongs to the initial data of domestic youth football running, which improves the vacancy of domestic reference materials for the development of theory and practice in this field. Through the research on the running distance analysis, aerobic and anaerobic intensity analysis, and running ability analysis of players in different positions of domestic top-level youth football players, this paper obtains the differences of each team and puts forward suggestions to some teams to better promote the development of youth football running ability.

## 3. Principle and Model of Dynamic Incremental Clustering Algorithm

In the clustering process, firstly, the density value of each data point *P*_*i*_(*i*=1,2,…, *m*) in dataset *D* is calculated, i.e., the overall density of the data space is modeled as the sum of the influence functions of all data points. Then, find the attraction point *O*_DensityMax_ with the largest local density, and take it as the center point of the first cluster. According to the adaptive density reachable radius *R*_Adap_, get the first density reachable cluster *C*_1_. Data structures commonly used in clustering algorithms include the data matrix and dissimilarity matrix, which are the measures of the distance between elements. Similarity is the premise and foundation of the clustering algorithm, and the basis of similarity measurement is distance. Hence, the study of distance is very important. Common distances include Euclidean distance, Mahalanobis distance, cosine similarity, weighted distance, etc. These distances have their own advantages and disadvantages, and how to choose the distance is very important to the clustering results. For large-scale dynamic incremental clustering algorithm clustering, when the dataset changes, it is necessary to consider completing the cluster update quickly. A fast compression method based on compressed set density accounting and central minimum inclusion ball technology can be introduced to compress large-scale datasets. Then, the degree of local synchronization is evaluated using and adopting the newly defined sequence parameters.

The process and purpose of model establishment are as shown in Figure 1 according to the research needs of the subject and the suggestions of experts.

Similarity is the basis of cluster analysis. How to construct similarity is very important. In the face of different data attributes, the calculation methods of similarity are different. Correlation coefficient is used to measure the similarity between two variables. The principle of canonical correlation analysis, the calculation method, and steps of typical components are studied. Transform *y* into two groups of variables with the largest correlation with X. Until the correlation of the two groups of variables is decomposed, the canonical component is selected to analyze the correlation of the two groups of variables through the canonical correlation coefficient and its significance test. The example shows that only the first canonical correlation coefficient can pass the significance test. The other two canonical correlation coefficients are significantly zero. Hence, the first pair of canonical components should be selected for analysis. The matrix composed of correlation coefficient is called the correlation coefficient matrix, and the angle similarity measure is also called cosine similarity. It is mainly used to measure the similarity between texts and is an important measure to detect text similarity. Distance is the basis for constructing similarity. Common distances include Euclidean, Markov, Chebyshev distance, etc. Distance has some well-known properties. If *d*(*x*, *y*) is the distance between two points *x* and *y*, the properties that hold are as follows:

1. Non-negativity, for *x*, *y* and *d*(*x*, *y*) ≥ 0, only *x*=*y* and *d*(*x*, *y*)=0
2. Symmetry, for all *x* and *y*, *d*(*x*, *y*)=*d*(*y*, *x*)

Triangular inequality, for all *x*, *y*, and *z*, has *d*(*x*, *y*) ≤ *d*(*y*, *z*)+*d*(*x*, *z*). Euclidean distance is defined as follows:

(1) $$\begin{array}{c} d\left(x,y\right)=\sqrt{\sum_{k=1}^{n}{\left(x_{k}-y_{k}\right)}^{2}}. \end{array}$$

*n* is the dimension, and *x*_*k*_ and *y*_*k*_ are the *x* attribute components of *y* and *k*, respectively. Euclidean distance is a common distance calculation formula in life, which is used to calculate the absolute distance between two numerical values in the Euclidean space. Without considering the correlation between components, multiple components reflecting a single feature will interfere with the results to keep the dimensions consistent. If the dimensions are different, we need to use the standardized Euclidean distance. By standardizing the data, the mean variance is equal. For example, in the sample set *X*, the mean value is *m*, and the standard deviation is *s*. Then, the standardized variable is expressed as (*x* − *m*)/*s*, and the standardized data is not affected by the dimensions.Minkowski distance is as follows:

(2) $$\begin{array}{c} d\left(x,y\right)={\left(\sum_{k=1}^{n}{\left|x_{k}-y_{k}\right|}^{r}\right)}^{1/r}. \end{array}$$

*r*=1, and Manhattan distance is the sum of the projections of line segments formed by two points on the fixed Cartesian coordinate system of the Euclidean space, which is mainly used in geometric metric space.

*r*=2, and Euclidean distance is used to describe the real distance between two points and is widely used.

*r*=*∞*, and supremum distance is the maximum distance between object attributes that belong to the hyperconvex measure.

The calculation formula of the membership degree and the iterative formula of the cluster center are derived by calculating the partial derivative of the Lagrange duality of the objective function. The whole process is a simple iteration. The objective function becomes the following:

(3) $$\begin{array}{c} J\left(X,U,C\right)=\sum_{i=1}^{c}\sum_{k=1}^{k}u_{ik}^{m}\left(x_{k}-c_{i}\right){\left(x_{k}-c_{i}\right)}^{T}. \end{array}$$

The objective function is the sum of the squares of the weighted distances from each data point to each cluster center, where *C* is the number of categories, *x*_*k*_ is the *k*^th^ sample, *c*_*i*_ is the cluster center of the *i*^th^ class, and *m* ∈ [1, +*∞*] is a weighted index. The larger the value of *m* is, the higher the fuzzy degree of classification is, and it is usually 2. If the membership degree of *u*_*ik*_ ∈ [0,1], *x*_*k*_ belonging to class *i*, and ∑_*i*=1_^*c*^*u*_*ik*_=1, ∀*k*=1,…, *K*, FCM is a process of continuously reducing the objective function. The objective function is solved by the Lagrange multiplier method, and the iterative formula for solving the membership degree is as follows:

(4) $$\begin{array}{c} u_{ik}=\frac{1}{\sum_{j=1}^{c}{\left(d_{ik}/d_{jk}\right)}^{2/\left(m-1\right)}}, \end{array}$$

where *d*_*ik*_ is the Euclidean distance between *k* samples and the *i* cluster center, and the iterative formula of the cluster center is as follows:

(5) $$\begin{array}{c} c_{i}=\frac{\sum_{K=1}^{K}u_{ik}^{m}x_{k}}{\sum_{j=1}^{K}u_{ij}^{m}}. \end{array}$$

The dataset is mapped to the feature space. After the dataset is mapped by the kernel function, the differences between different categories are increased, and the linearly nonseparable dataset is changed into linearly separable data. In this way, clustering can be carried out in a high-dimensional space. Adding the kernel function has a stronger learning ability and generalization ability. The commonly used kernel functions include the polynomial kernel function and Gaussian kernel function. The specific forms are as follows:

(6) $$\begin{array}{c} K\left(x_{i},x_{j}\right)={\left(x_{i}\cdot x_{j}+1\right)}^{p}. \end{array}$$

The polynomial kernel function is a global kernel function with poor locality, in which *p* is the highest degree of polynomial function, and *p* is not easy to be too large. Otherwise, the elements of the kernel matrix will tend to infinity, generally taking 2.

(7) $$\begin{array}{c} K\left(x_{i},x_{j}\right)=\exp\left(-\frac{{\left\|x_{i}-x_{j}\right\|}^{2}}{2\delta^{2}}\right). \end{array}$$

The Gaussian kernel function is a kernel function with strong locality. *σ* is the bandwidth of the Gaussian kernel function, which is equal to 2 by default, and its extrapolation ability decreases with the increase of parameter *σ*.

Let *x*_*i*_ and *x*_*j*_ become Φ(*x*_*i*_) and Φ(*x*_*j*_) after kernel function mapping. Then, the formula of the Euclidean distance of elements in feature space is as follows:

(8) $$\begin{array}{c} d\left(x_{i},x_{j}\right)=\Phi \left(x_{i}\right)-\Phi \left(x_{j}\right)=\sqrt{k\left(x_{i},x_{i}\right)-2k\left(x_{i},x_{j}\right)+k\left(x_{j},x_{j}\right)}. \end{array}$$

Assuming that the dataset is {*x*_1_, *x*_2_,…, *x*_*n*_}, the formula for defining the average distance of elements is as follows:

(9) $$\begin{array}{c} \overset{-}{d}=\frac{1}{C_{n}^{2}}\sum_{i=1}^{n}\sum_{j=1}^{i}d\left(x_{i},x_{j}\right). \end{array}$$

*n* is the number of samples, *C*_*n*_^2^ is all the optional combinations of two randomly selected samples, and *d*(*x*_*i*_, *x*_*j*_) is the distance from *x*_*i*_ to *x*_*j*_.

Let $\overset{-}{x}$ data be {*x*_1_, *x*_2_,…, *x*_*n*_}. Then, their variance calculation formula is as follows:

(10) $$\begin{array}{c} \text{VAR}\left(s^{2}\right)=\frac{1}{n}\sum_{i=1}^{n}{\left(x_{i}-\overset{-}{x}\right)}^{2}. \end{array}$$

Among them, $\overset{-}{x}$ is the average distance, and its calculation formula is $\overset{-}{x}=1/n\sum_{i=1}^{n}x_{i}$.

## 4. The Realization of the Model of Football Trainer's Running Ability Mining

### 4.1. Running Ability Mining of Football Trainers Based on Dynamic Incremental Clustering Algorithm

Based on the dynamic incremental clustering algorithm, this paper hopes to assist coaches to find the technical and tactical categories of small players. At the same time, the clustering samples are three-dimensional acceleration indicators. There is no problem of different density caused by the wide variety of clustering sample data. Methods to reduce time complexity include making full use of existing information and using a certain data structure. For the two scenarios used by different priority queues, the map is sorted according to the value of the map. At the same time, sort the collection of some elements. At this time, you can define a class for these elements. Therefore, the k-means algorithm in the clustering algorithm is the most appropriate. However, because of the large amount of training running data and real-time change and update, the complexity of the algorithm should not be too high. Many classical clustering algorithms are difficult to meet this. Therefore, based on the k-means algorithm, this paper adopts the dynamic incremental clustering algorithm based on the center point, inherits the existing clustering results, avoids the problem of reclustering all the data every time the data is updated, and effectively reduces the complexity of the algorithm. In modern football matches, the requirements for forwards are higher. In addition to having efficient scoring ability, the ability to connect with avant-garde players in attack, involve defensive players, and create scoring opportunities for avant-garde players should also be improved accordingly. Therefore, we see more goals from avant-garde players, which are related to the running of avant-garde players in the game.

Football is a sport that requires a good combination of technology and speed. The technology of football should have running speed as the premise and guarantee. Football players should do a lot of actions, such as starting, sharp turn, sudden stop, changing direction, changing speed, and turning around, which requires excellent instantaneous speed, acceleration, braking speed, and maximum speed. However, the existing training methods are judged by coaches' naked eyes and experience. Hence, it is difficult to know its essence deeply. Each athlete's training assistant keeps the rubber strip at approximately the same tensile tension during each 60-meter run to obtain the overspeed effect of resistance. Based on the dynamic incremental clustering algorithm, when the training assistant and the test athlete run in the same direction, the distance between them is roughly the same. The assistant accelerates with the acceleration of the athlete, and the 60-meter process should always keep accelerating. Although in terms of running distance, the data of forwards and defenders are equal, forwards are in an active running state most of the time. Under normal circumstances, they always interfere with 1–2 defenders. Therefore, excellent running ability is essential for forwards. The basic idea of the application of dynamic incremental clustering algorithm in athletes' running ability mining is as follows: cluster the weighted accelerations of 10 players within 5 minutes before training with the classical K-means clustering algorithm and preliminarily define the categories of athletes' running ability. Actually, according to the needs of coaches, the young players are divided into three categories: active, steady, and negative. Hence, *k* takes a value of 3. On this basis, after every 5 minutes, the increment of acceleration information of each training player is obtained, and the increment data is clustered until the end of training. In the dynamic incremental clustering algorithm, we can see that with the addition of incremental data, although the incremental clustering algorithm updates the original clustering locally or globally, as this paper focuses on the comprehensive running ability of young players in the whole game, it is finally necessary to globally weigh several incremental clustering information before the final clustering result is obtained.

### 4.2. Experimental Results and Analysis

The evaluation of clustering quality lies in the following two aspects: the internal compactness of clusters and the distance between clusters as far as possible, i.e., intraclass differences and interclass differences. The larger or smaller the threshold, the more outliers and the impact on intraclass and interclass, as shown in Table 1.

It can be seen from Table 1 that the comparison of quality indicators of each cluster can be seen, *ε*. When the value is 1.2 g, the clustering quality is the highest. According to the calculation formula of 1G = 9.8 m/s^2^, it is equivalent to the acceleration level of about 10 m/s^2^ for each cluster, which is more in line with the wide difference of sports types in the actual running of football.

This paper analyzes the data of a football game between teenagers. According to the analysis, the actual time of football match is longer than before. The average game time is 94–99 minutes. The actual game time has increased from 52 to 56 minutes in 1990 to more than 60 minutes now. The average actual time of each game in this world cup is 66.95 min. The running forms of players in fierce competition can be divided into three types: slow running (60–70% maximum heart rate), medium running (80–90% maximum heart rate), and fast running (90–100% maximum heart rate). The running form of defenders is shown in Table 2.

From Table 2, it can be seen that in each game of the draw, the slow running time of defenders is more than 50 min, accounting for the largest proportion. The ratio of middle-speed running and fast running is equal, with the time being more than 4.4 min. In the competition, the distance of slow running is at least 5.4 km. The distance of middle-speed running is 1–2 km, the distance of fast running is more than 2 km, and the fast-running distance of fullbacks is more than that of central defenders. In addition, in terms of players' speed, the average fastest speed of defenders reached 25.56 km/h, and some players reached more than 27 km/h. The basic value model represents the basic value of the selected evaluation index, and it is also the embodiment of the basic characteristics of athletes' running ability in different positions, as shown in Table 3.

The statistical analysis of the running distance of avant-garde players shows that the total running distance, running distance with the ball, and running distance without the ball of avant-garde players are more than those of defenders. The average running distance of each game is between 10 and 12 km, and the most in the 90-minute game is 13.26 km. Some of the players, such as Harvey, Schweinsteiger, and Hedila, have maintained a high level of physical fitness throughout the game, The average total running distance of each game is more than 10 km. According to the player's position and offensive and defensive ability, the offensive midfield, such as the front waist and the winger, has relatively more running distance with the ball, and the defensive midfield with the back waist has more running distance without the ball. These two data are also higher than those for the defender. The statistical table of running distance of avant-garde players is shown in Table 4.

From Table 4, it can be seen that in terms of the time and distance of middle-speed running and fast running, avant-garde players have higher requirements than defenders, among which, the fast-running time is equal, however, the distance is more than the middle-speed running distance. Players who play a central role in each team have shown a high level in middle-speed running and fast running, such as Harvey, Alonso, Schweinsteiger, and other players, who are the planners of the team's attack and the masters of the game rhythm. The method of establishing comprehensive evaluation criteria also adopts the percentile method, which is the same as the establishment of single evaluation criteria, as shown in Table 5.

In the first half of the game, if the shooting technique is not consistent, then the players will be unable to play the ball in the first half, and if the shooting technique is not consistent, the players cannot even stop the ball in the second half. If there is a phenomenon of slow cooperation in the first half, the players cannot even play the ball in the second half. The main reason is that the students' physical quality cannot meet the requirements of the competition and cannot bear fierce confrontation. To further understand the physical quality level of students and facilitate quality training in the future, we have specially made a series of physical fitness tests, and the results are shown in Table 6.

From Table 6, it can be seen that the results of the above physical fitness tests are really somewhat promising. Students with this level of physical fitness will suffer from dizziness, cramps, vomiting, etc., even in normal training, and it takes a long time to recover after practice. To improve the ability of self-protection in fierce confrontation, a set of methods of quality exercises are developed according to their current physical condition. These methods mainly include speed, strength, endurance, bounce, sensitivity, and flexibility.

Using the methods of expert screening and logical analysis, this experiment evaluates and tests the score percentage of the existing forwards, midfielders, and defenders and establishes the evaluation index of athletes' running ability in different positions. The distribution of this experiment was compared three times, and the experimental results are shown inFigure 2–4.

From Figure 2 to Figure 4, it can be seen that sprint and high-speed running are very important for the three positions. From the above results, combined with the suggestions of statistical experts, this study decided to preliminarily establish the index with a frequency of more than 60%. During the period when the time index is 40, the average score of the forward is 65.3%, the average score of the avant-garde is 67.6%, and the average score of the guard is 64.8%. Among them, the avant-garde has the highest proportion, and the evaluation indicators are sprint, high-speed running, and total running distance. The evaluation indexes of avant-garde are sprint, high-speed running, total running distance, and medium speed running. The evaluation indexes of guards are sprint, high-speed running, and total running distance.

In this experiment, the percentile method was used to formulate the evaluation criteria of individual indicators, which were divided into five grades, namely, first-class, middle-class, lower-class, and the corresponding percentile intervals were 10%, 15%, 50%, 15%, and 10%, respectively. The experimental results were compared in two experiments, as shown in Figure 5.

It can be seen from Figure 5 that the significance of the formulation of single evaluation criteria is that it can evaluate the single indicators of athletes in different positions. For example, forward athletes can compare the test results of their different indicators with the evaluation criteria to obtain the grades of various indicators, so as to find their advantages and disadvantages running indicators and to provide reference and reference for the scientific monitoring of training and competition. The comprehensive evaluation standard is a comprehensive evaluation of the running ability of athletes in different positions, which can reflect the comprehensive running ability and level of athletes. It is the core content and method of competition physical fitness evaluation.

## 5. Conclusions

In this paper, the dynamic incremental clustering algorithm is applied to the classification of football training athletes' running ability. It can not only effectively mine and classify football training athletes' running but also avoid the surge of calculation caused by the surge of dynamic data during running. It can realize the clustering of large datasets generated by football running, which is more objective, intelligent, and significant. According to scientific procedures and methods, this study established the model and standard of Chinese elite women football players' running ability in competition, and the validity of the model verified by the standard identification method was 0.83. It indicated that this evaluation model was highly efficient. In a team, the players' health and abundant physical fitness are the prerequisites for the team to maintain a high level and stable performance for a long time. The players of international level take part in 60–70 matches every season. In such a fierce and tense season, how to make the players' running ability meet the needs of matches is one of the training focuses that coaches attach great importance to today. The data source is wireless acceleration sensor data, which will inevitably produce noise data during running and transmission. It will affect the clustering results of this paper to a certain extent. In the next step, to make the original dataset more intelligent and accurate, we will consider denoising the original data. This model is rich in data, and the testing methods and procedures are basically standardized. It can be used as a yardstick for the running ability of Chinese elite women football players in a certain period and scope. At the same time, the procedures and methods established by this model can provide reference for other related studies.

## Figures and Tables

**Figure 1:** Running ability model of football match.

**Figure 2:** Selection results of evaluation index experts.

**Figure 3:** Selection results of evaluation index experts.

**Figure 4:** Selection results of evaluation index experts.

**Figure 5:** Grade evaluation standard of single evaluation index.

**Table 1:** Intraclass and interclass differences of different clustering results when threshold *ε* is input.

Threshold *ε*	Maximum diameter in cluster	Minimum cluster diameter	Average cluster diameter	Maximum difference between clusters	Minimum difference between clusters	Average value of difference between clusters
0.6	2.851	2.542	2.674	2.671	2.354	2.467
0.7	2.842	2.541	2.652	2.686	2.361	2.484
0.8	2.872	2.535	2.633	2.714	2.386	2.551
1	2.821	2.531	2.662	2.622	2.312	2.461
1.1	2.814	2.531	2.624	2.762	2.403	2.683

**Table 2:** Statistics of defender's running formballplayer.

Ballplayer	Average per game						
	Slow running time (min)	Slow running distance (km)	Medium running time (min)	Medium distance (km)	Fast-running time (min)	Fast-running distance (km)	90 min fastest running speed/(km/h)
Ramos	50.56	5.52	5.28	1.48	6.42	2.82	26.71
Kapu devilla	53.28	5.84	5.01	1.47	5.42	2.46	26.08
Simon van der Meer	52.41	5.91	5.81	1.71	6.61	2.38	26.23
Fusile	51.52	5.42	4.62	1.35	6.22	2.61	24.82
Mattheiszen	55.16	5.92	4.82	1.38	4.66	1.88	26.21

**Table 3:** List of basic value models of evaluation indicators.

Movement form	Forward	Midfielder	Guard
Sprint run	254	161	134
High-speed running	551	462	377
Medium-speed running	677	343	356
Total distance	569	608	626

**Table 4:** Statistical table of running distance of avant-garde players.

Ballplayer	Location	Competition time/min	Average per game			Maximum running distance of 90 min/km
			Total running distance/km	Running distance of the ball/km	No ball running distance/km	
Harvey	Qianyao	635	11.45	5.55	3.58	12.31
Sneijder	Qianyao	651	10.46	4.24	3.86	10.81
Sergi Busquets Burgos	Small of the back	632	10.21	4.23	3.92	10.83
Khedira	Small of the back	607	12.21	4.74	4.62	12.26

**Table 5:** List of comprehensive evaluation grade standards.

	Forward	Midfielder	Guard
Superior	>17.7	>14.2	>17.3
Medium and superior	17.7–15	14.2–12.7	17.3–13.4
Secondary	15.8–10.2	12.6–7.7	13.5–6.8
Middle and lower-class	11–8.3	7.8–6.3	6.7–3.4
Inferior	<8.1	<6.3	<3.4

**Table 6:** Comparison between students' physical fitness and sports standards.

Speed	Project	30 m	50 m	100 m
	Standard	3″8	6″	12″2
	Selected students	4″1	6″3	12″6

Endurance	Project	1000 m	1500 m	3200 m
	Standard	3′04′	5′01″	12′03″
	Selected students	3′14″	5′24″	14′16″

Force	Project	Pull-ups (pieces)	Throw a solid ball (M)	50 kg weight-bearing station squat (times/minute)
	Standard	24	13.52	21
	Selected students	15	11.22	14

## Data Availability

The data used to support the findings of this study are included within the article.
